# Analysis on the Effect of the Rehabilitation Intervention-Centered Targeted Nursing Model on the Cardiac Function Recovery and Negative Emotions in Patients with Acute Myocardial Infarction

**DOI:** 10.1155/2022/1246092

**Published:** 2022-02-24

**Authors:** Rong Wang, Gongxiang Duan, Huilan Xu, Yuanyuan Wu, Yinhua Su, Jianzhi Li, Li Liao, Daqi Liao

**Affiliations:** ^1^Xiangya School of Public Health, Central South University, Changsha, Hunan 410001, China; ^2^School of Nursing, University of South China, Hengyang, Hunan 421001, China; ^3^Wuxi Mental Health Center, Wuxi 214000, China

## Abstract

Rehabilitation intervention which refers to the functional training by caregivers with the aid of specialized nursing techniques and the progressive promotion of patients' training initiative, with the purpose of improving mobility and quality of life, is of great significance. The purpose of the study was to investigate the effect of the rehabilitation intervention-centered targeted nursing model on the cardiac function recovery and negative emotions in patients with acute myocardial infarction (AMI). A total of 120 AMI patients admitted to our hospital between January 2019 and January 2020 were selected as the study subjects and randomly divided into group A (*n* = 60) and group B (*n* = 60), in which the group B patients received routine nursing combined with rehabilitation intervention, while based on the treatment in group B, the patients in group A underwent rehabilitation intervention-centered targeted nursing model. Then, the cardiac function indexes, negative emotion score, levels of risk factors for heart failure, complication rate (CR), and the quality of life (QOL) of the patients were compared between the two groups. The cardiac function indexes of the patients after nursing in group A were significantly better than those in group B (*P* < 0.001); the negative emotion scores of the patients after nursing in group A were significantly lower than those in group B (*P* < 0.001); the levels of risk factors for heart failure of the patients after nursing in group A were significantly lower than those in group B (*P* < 0.001); the CR of the patients in group A at 15 d and 30 d after admission was significantly lower than that in group B (*P* < 0.05); the QOL scores of the patients after nursing in group A were significantly higher than those in group B (*P* < 0.001). Rehabilitation intervention-centered targeted nursing model can optimize cardiac function, weaken the levels of risk factors for heart failure, reduce the incidence of complications, improve psychological conditions, and enhance the quality of life in AMI patients, which is worthy of application and promotion in clinical practice.

## 1. Introduction

The majority of AMI patients usually presents with myocardial ischemia and hypoxia, declined cardiac function, and impaired respiratory system, further leading to their weakened mobility; therefore, rehabilitation intervention which refers to the functional training by caregivers with the aid of specialized nursing techniques and the progressive promotion of patients' training initiative, with the purpose of improving mobility and quality of life, is of great significance [1–3]. However, current studies on the rehabilitation intervention for AMI patients in clinical practice have revealed that, due to the twin stressors of physical and psychological conditions, patients have low compliance with rehabilitation training; besides, the routine nursing model is less targeted and cannot relieve patients' negative emotions, so it has relatively limited effect on facilitating rehabilitation [4–7]. AMI patients' great suffering of severe pain at the onset of the disease combined with the oppressive hospital environment can result in their heavy psychological burdens, which may further aggravate or eventually come with an extremely obvious tendency of anxiety and depression, greatly hindering the progress of rehabilitation. At present, targeted nursing has become one of the focuses of clinical concern, and it considers patients' subjective complaints and actual conditions as the implementation basis of nursing measures, with the advantages of high pertinence and personalized services. Based on this, in order to investigate the effect of the rehabilitation intervention-centered targeted nursing model on AMI patients, a total of 120 AMI patients admitted to our hospital between January 2019 and January 2020 were selected as the study subjects, and the study results are summarized as follows.

## 2. Materials and Methods

### 2.1. General Information

A total of 120 AMI patients admitted to our hospital between January 2019 and January 2020 were selected as the study subjects and randomly divided into group A (*n* = 60) and group B (*n* = 60). There were no significant differences in the general information of the patients between the two groups (*P* > 0.05), with research significance, as detailed in Table 1.

### 2.2. Inclusion Criteria

The inclusion criteria were as follows: (1) patients and their family members were informed of the purpose and process of the study and signed informed consent. (2) Patients met the AMI diagnostic criteria made by the American Heart Association [8, 9]. (3) Patients had the onset within twelve hours. (4) Patients' Killip classification of cardiac function was below IV. (5) This study was approved by the hospital.

### 2.3. Exclusion Criteria

The exclusion criteria were as follows: (1) patients had other organic diseases or complications such as pulmonary edema. (2) Patients had mental disorders or could not communicate with others. (3) Patients had lumbar fracture.

### 2.4. Methods

The group B patients received routine nursing combined with rehabilitation intervention, and the specific steps were as follows. (1) Nursing staff should pay much attention to the changes of patients' sign data to check whether there were signs of deterioration and provide patients with routine diet and medication guidance. (2) Nursing staff should ask the patients to lie in bed for a rest and provide physical nursing by the way of wiping patients' skin to perform the passive activity within one week of onset. After one week, the patients were encouraged to get up by themselves and perform stretching in semireclining positions. After two weeks, the patients were instructed to get out of bed to do some exercises, such as walking, and their walking time could be prolonged with the increase of rehabilitation intervention, and nursing staff should pay much attention to the occurrence of adverse reactions in patients.

Based on the treatment in group B, the patients in group A were given extra rehabilitation intervention-centered targeted nursing model, and the specific steps were as follows. (1) Nursing staff should increase their own empathy to keep close to patients' mental status and timely carry out psychological counseling. Besides, in order to improve patients' cooperation with the rehabilitation, nursing staff should frequently tell patients the positive significance of rehabilitation training, adopt integrating or target systems to promote their motor initiative, and timely give patients encouragement and rewards after they reached their small goals. At the same time, when patients were undergoing rehabilitation training, nursing staff should explain the knowledge related to the disease timely and play some soothing music to relieve their anxiety and restlessness. (2) Before the initiation of nursing care, nursing staff should comprehensively grasp patients' clinical data, increase the frequency of communication, listen to their subjective appeal, and adjust nursing plans at any time according to patients' specific demands and actual conditions, so as to make the rehabilitation intervention program personalized. (3) Nursing staff should carry out rehabilitation within 24 hours of patients' onset by the way that patients changed their supine positions to semireclining positions which were then kept for half an hour, and then the patients returned to their original supine positions with the help of nursing staff. Such position-changing exercises were required to be performed more than 3 times per day. After one day of patients' onset, nursing staff should tell patients the positive role of getting up from bed on their own to arouse their willingness to get up actively and help them perform physical stretching in semireclining positions. At two days after patients' onset, nursing staff should ask patients to carry out sitting training on bed and strengthen the exercise with enhanced rehabilitation intervention. At three days after patients' onset, the patients were asked to get out of the bed to stand for no less than 10 minutes per day, and additionally, they were encouraged to walk, and after four days, the patients should intensify the training in walking by prolonging walking distance [10–13]. (4) Nursing staff should encourage patients' family members to pay much attention to patients, effectively exerting the dual functions of professional nursing and family nursing.

### 2.5. Observation Indexes

1. Levels of risk factors for heart failure: the levels of angiotensin II (Ang II), aldosterone (ALD), and B-type natriuretic peptide (BNP) were compared between the two groups
2. CR: the rate of complications including arrhythmia and heart failure was compared between the two groups at 1 d (*T*_1_), 15 d (*T*_2_), and 30 d (*T*_3_) after admission
3. Cardiac function indexes: the left ventricular end-systolic dimension (LVESD), left ventricular end-diastolic dimension (LVEDD), left ventricular ejection fraction (LVEF), and early/late diastolic peak velocity of the left atrioventricular valve (E/A ratio) before and after nursing intervention were compared between the two groups
4. Negative emotion score: the negative emotions of the patients were evaluated by the self-rating anxiety scale (SAS) and the self-rating depression scale (SDS), and higher scores indicated severer negative emotions in patients
5. QOL: the QOL was evaluated by the QOL-C30 scale, whose items included emotional function, physical function, social function, role function, and cognitive function, and higher scores indicated better QOL

### 2.6. Statistical Treatment

The selected data processing software for this study was SPSS 20.0, and software selected to draw the pictures was GraphPad Prism 7 (GraphPad Software, San Diego, USA). Measurement data were tested by *t*-test, and enumeration data were tested by *X*^2^ test. The differences had statistical significance when *P* < 0.05.

## 3. Results

### 3.1. Comparison of Cardiac Function Indexes between the Two Groups

After nursing, the LVESD and LVEDD levels in group A were significantly lower than those in group B (*P* < 0.001), and the LVEF level and E/A ratio in group A were significantly higher than those in group B (*P* < 0.001), as shown in Table 2.

### 3.2. Comparison of Negative Emotion Scores between the Two Groups

After nursing, the negative emotion scores in group A were significantly lower than those in group B (*P* < 0.001), as shown in Table 3.

### 3.3. Comparison of the Levels of Risk Factors for Heart Failure between the Two Groups

The levels of risk factors for heart failure after nursing in group A were significantly lower than those in group B (*P* < 0.001), as shown in Table 4.

### 3.4. Comparison of CR between the Two Groups

The CR in group A at *T*_2_ and *T*_3_ was significantly lower than that in group B (*P* < 0.05), as shown in Figures 1 and 2.

### 3.5. Comparison of the QOL after Nursing between the Two Groups

The QOL scores after nursing in group A were significantly higher than those in group B (*P* < 0.001), as shown in Figure 3.

## 4. Discussion

AMI patients' great suffering of severe pain at the onset of the disease combined with the oppressive hospital environment can result in their heavy psychological burdens, which may further aggravate or eventually come with an extremely obvious tendency of anxiety and depression, greatly hindering the progress of rehabilitation [14–17]. Routine nursing care mainly focuses on the clinical efficacy of rehabilitation intervention, and nursing staff usually lay emphasis on the completion degree of functional training tasks and ignore timely psychological counseling, and thus, patients' depression cannot be addressed, and rehabilitation effect remains unsatisfactory. Better intervention effect can be achieved by enhancing the frequency of communication with patients, listening to their subjective appeals, and developing more targeted and personalized nursing measures for them [18–22]. The majority of AMI patients usually presents with myocardial ischemia and hypoxia, declined cardiac function, and impaired respiratory system, further leading to their weakened mobility; therefore, rehabilitation intervention which refers to the functional training by caregivers with the aid of specialized nursing techniques and the progressive promotion of patients' training initiative, with the purpose of improving mobility and quality of life, is of great significance.

In this study, the negative emotion scores of the patients in group A after nursing were significantly lower than those in group B (*P* < 0.001) because nursing staff alleviates patients' anxiety and depression by introducing the knowledge related to the disease in detail and actively responding to the problems raised by the patients, so patients' adverse emotions are effectively relieved. Due to more positive emotions, an increased initiative to perform rehabilitation training, and the combination with rehabilitation intervention in the early stage of the disease in group A, the cardiac function indexes as well as the levels of risk factors for heart failure in group A after nursing were significantly better than those in group B (*P* < 0.001), and the CR at 15 d and 30 d after admission in group A was significantly lower than that in group B (*P* < 0.05), indicating that nursing can greatly improve patents' hypoxia tolerance and effectively promote the recovery of cardiac function and exercise capacity, with more desirable recovery effect.

## 5. Conclusion

Moreover, as a result of increased frequency of communication with patient's family members and better mastery of rehabilitation knowledge, the QOL scores of the patients in group A after nursing were significantly higher than those in group B (*P* < 0.001), and the functional scores in all aspects of the patients in group A were better than those in group B, confirming the positive effect of the targeted nursing intervention. Scholar Tracy Sue in her study pointed out that the scores of emotional function, physical function, social function, role function, and cognitive function in the research group, in which the patients receive the functional rehabilitation-centered targeted nursing model, are 86.61 ± 3.22 points, 75.20 ± 5.02 points, 77.89 ± 4.21 points, 82.31 ± 3.41 points, and 76.11 ± 4.90 points, respectively, which are all significantly higher than those in the reference group where the patients underwent routine rehabilitation intervention (*P* < 0.001), indicating that patients in the research group have a better quality of life and recovery [23]. Her study results are in line with the findings concluded in our study.

In conclusion, rehabilitation intervention-centered targeted nursing model can effectively enhance cardiac function and relieve negative emotions of AMI patients, which is worthy of application and promotion in clinical practice. In the future, we need more cases to ensure the reliability of the experimental results. Our experiment still has many limitations.

## Figures and Tables

**Figure 1:** Comparison of the incidence of arrhythmia between the two groups. Note: the abscissa represented 1 d (*T*_1_), 15 d (*T*_2_), and 30 d (*T*_3_) after admission. The incidence of arrhythmias at *T*_1_ was 66.7% (40/60) in group A and 70.0% (42/60) in group B. The incidence of arrhythmias at *T*_2_ was 40.0% (24/60) in group A and 60.0% (36/60) in group B. The incidence of arrhythmias at *T*_3_ was 30.0% (18/60) in group A and 53.3% (32/60) in group B. ^*∗*^*P* < 0.05.

**Figure 2:** Comparison of the incidence of heart failure between the two groups. Note: the abscissa represented 1 d (*T*_1_), 15 d (*T*_2_), and 30 d (*T*_3_) after admission. The incidence of heart failure at *T*_1_ was 40.0% (24/60) in group A and 40.0% (24/60) in group B. The incidence of heart failure at *T*_2_ was 10.0% (6/60) in group A and 30.0% (18/60) in group B. The incidence of heart failure at *T*_3_ was 1.7% (1/60) in group A and 16.7% (10/60) in group B. ^*∗*^*P* < 0.05.

**Figure 3:** Comparison of the QOL after nursing between the two groups ($\bar{x}\pm s$, points). Note: the abscissa represented emotional function, physical function, social function, role function, and cognitive function. The emotional function scores were 86.21 ± 4.22 points in group A and 75.02 ± 5.41 points in group B. The physical function scores were 74.20 ± 5.21 points in group A and 69.10 ± 5.32 points in group B. The social function scores were 77.81 ± 3.02 points in group A and 67.23 ± 3.00 points in group B. The role function scores were 80.12 ± 2.41 points in group A and 70.23 ± 3.16 points in group B. The cognitive function scores were 76.20 ± 5.20 points in group A and 69.10 ± 3.00 points in group B. ^#^*P* < 0.001.

**Table 1:** Comparison of general information between the two groups.

Group	Group A (*n* = 60)	Group B (*n* = 60)	*X* ^2^/*t*	*P*
Gender			0.038	0.845
Male	40	41		
Female	20	19		

*Age (years)*				
Age range	32–74	33–74		
Average age	51.21 ± 6.20	51.23 ± 6.21	0.018	0.986
Hypertension	32	33	0.034	0.855
Cerebral infarction	12	13	0.051	0.822
Diabetes mellitus	25	24	0.035	0.853

*Infarction location*				
Anterior wall	25	24	0.035	0.853
Inferior wall	18	18	0.000	1.000
Side wall	10	8	0.261	0.609
Others	7	10	0.617	0.432

*Killip classification*				
I	26	27	0.034	0.854
II	22	20	0.147	0.702
III	12	13	0.051	0.822

**Table 2:** Comparison of cardiac function indexes between the two groups $\left(\bar{x}\pm s\right)$.

Types	Group A		Group B		*t*	*P*
LVESD (mm)	Before nursing	55.21 ± 3.56	Before nursing	55.23 ± 4.01	0.029	0.977
	After nursing	47.12 ± 3.25	After nursing	52.23 ± 3.58	8.186	≤0.001
	*t*	13.000	*t*	4.323		
	*P*	≤0.001	*P*	≤0.001		
LVEDD (mm)	Before nursing	62.12 ± 4.56	Before nursing	62.23 ± 4.65	0.131	0.896
	After nursing	50.23 ± 3.98	After nursing	58.11 ± 3.54	11.459	≤0.001
	*t*	15.217	*t*	5.461		
	*P*	≤0.001	*P*	≤0.001		
LVEF (%)	Before nursing	45.65 ± 4.01	Before nursing	45.78 ± 4.02	0.177	0.860
	After nursing	59.12 ± 5.78	After nursing	52.89 ± 5.79	5.899	≤0.001
	*t*	14.832	*t*	7.813		
	*P*	≤0.001	*P*	≤0.001		
E/A ratio	Before nursing	0.81 ± 0.21	Before nursing	0.82 ± 0.20	0.267	0.790
	After nursing	2.01 ± 0.32	After nursing	1.35 ± 0.36	10.614	≤0.001
	*t*	24.285	*t*	9.969		
	*P*	≤0.001	*P*	≤0.001		

**Table 3:** Comparison of negative emotion scores between the two groups ($\bar{x}\pm s$, points).

Group	SDS		SAS		
	Before nursing	After nursing	Before nursing		After nursing
Group A	50.12 ± 5.32	30.26 ± 2.12	56.15 ± 5.30	35.11 ± 2.87	
Group B	50.32 ± 5.56	38.45 ± 3.68	56.35 ± 4.89	43.12 ± 4.85	
*t*	0.201	14.938	0.215	11.010	
*P*	0.841	≤0.001	0.831	≤0.001	

**Table 4:** Comparison of the levels of risk factors for heart failure between the two groups ($\bar{x}\pm s$, pg/ml).

Types	Group A		Group B		*t*	*P*
Ang II	Before nursing	160.21 ± 13.56	Before nursing	161.20 ± 13.25	0.404	0.687
	After nursing	110.20 ± 10.55	After nursing	130.35 ± 10.58	10.446	≤0.001
	*t*	22.547	*t*	14.093		
	*P*	≤0.001	*P*	≤0.001		
ALD	Before nursing	172.41 ± 15.45	Before nursing	172.42 ± 15.56	0.004	0.997
	After nursing	132.58 ± 10.50	After nursing	156.32 ± 12.59	11.217	≤0.001
	*t*	16.516	*t*	6.231		
	*P*	≤0.001	*P*	≤0.001		
BNP	Before nursing	565.21 ± 74.21	Before nursing	566.50 ± 75.41	0.094	0.925
	After nursing	160.25 ± 30.58	After nursing	240.65 ± 42.59	11.878	≤0.001
	*t*	39.081	*t*	29.144		
	*P*	≤0.001	*P*	≤0.001		

## Data Availability

The datasets used and/or analyzed during the current study are available from the corresponding author upon reasonable request.
